The article "Effect and Mechanism of lncRNA CERS6-AS1 on the Biological Behavior of Prostate Cancer Cell" was retracted in 2023. Reasons: signs of a paper mill; suspected computer-generated content; unreliable results or conclusions; concerns about the data.

# Effect and Mechanism of lncRNA CERS6-AS1 on the Biological Behavior of Prostate Cancer Cell

**DOI:** 10.1155/2022/9292538

**Published:** 2022-06-06

**Authors:** Fu Huang, Li Quan Zhou

**Affiliations:** Department of Urology, The Second Affiliated Hospital of Guangxi Medical University, China

## Abstract

**Objective:**

To investigate the effect of long noncoding RNA (lncRNA) CERS6 antisense RNA1 (CERS6-AS1) on the biological behavior of prostate cancer cells DU145 and its mechanism.

**Methods:**

RT-PCR was used to detect the relative level of CERS6-AS1 and miR-16-5p in prostate cancer tissues, adjacent tissues, prostate cancer cells DU145, and human normal prostate epithelial cells RWPE-1. DU145 cells were divided into control group, si-CERS6-AS1 group, si-NC group, miR-16-5p mimic group, miR-NC group, and si-CERS6-AS1+miR-16-5p inhibitor group. And CCK-8 method and colony formation test was applied to detect cell proliferation ability, flow cytometry was selected to calculate cell apoptosis, and scratch healing test was employed to assess cell migration ability. Western blot was determined to detect high mobility protein A2 (HMGA2) expression. RT-PCR and dual-luciferase reporter experiments were used to analyze the targeting relationship among CERS6-AS1, miR-16-5p, and HMGA2.

**Results:**

Compared with the adjacent tissues, the relative level of CERS6-AS1 in prostate cancer tissue was increased (*P* < 0.05), and the relative level of miR-16-5p was decreased (*P* < 0.05). Compared with RWPE-1 cells, the relative level of CERS6-AS1 in DU145 cells was increased (*P* < 0.05), and the relative level of miR-16-5p was decreased (*P* < 0.05). Compared with the control group and the si-NC group, the HMGA2 protein expression, the colony formation number, and the scratch healing rate of DU145 cells in the si-CERS6-AS1 group and the miR-16-5p mimic group were reduced (*P* < 0.05), and the relative level of miR-16-5p and the proliferation inhibition rate and apoptosis were increased (*P* < 0.05). miR-16-5p is specifically bound to CERS6-AS1 and HMGA2, respectively. Compared with the si-CERS6-AS1 group, the HMGA2 protein expression, the colony formation number, and the scratch healing rate of DU145 cells in the si-CERS6-AS1+miR-16-5p inhibitor group were increased (*P* < 0.05), and the cell proliferation inhibition rate and apoptosis rate were reduced (*P* < 0.05).

**Conclusion:**

Silencing CERS6-AS1 can inhibit the proliferation and migration of prostate cancer cell DU145 and induce cell apoptosis, the mechanism is related to the regulation of the miR-16-5p/HMGA2 axis.

## 1. Introduction

Prostate cancer is the second most common cancer among men in the world. In 2021, there were about 1.3 million new cases of prostate cancer and about 359000 deaths [1]. Androgen deprivation therapy through surgery or drugs is the standard first-line treatment for patients with metastatic prostate cancer, but most patients will develop castration resistant prostate cancer within 2~3 years, and their survival status is still very poor [1]. Therefore, further exploring the regulatory mechanism of prostate cancer progression is of great significance to develop new treatment strategies.

Long chain noncoding RNA (lncRNA) is a class of RNA molecules with transcripts longer than 200 NT, which can regulate gene expression at different levels. It has been found that lncRNA can interact with microRNA (miRNA), participate in regulating the expression of target mRNA, and play an important role in tumorigenesis and metastasis [2, 3]. There is evidence that the upregulated expression of CERS6 antisense RNA1 (CERS6-AS1) can predict the poor prognosis in patients with liver cancer [4].

Overexpression of CERS6-AS1 in breast cancer can promote the proliferation of breast cancer cells and inhibit cell apoptosis [5]. However, the role of CERS6-AS1 in prostate cancer has not been reported. miR-16-5p is a tumor suppressor. Studies have found that miR-16-5p can induce the decline of prostate cancer cell viability and G0/G1 cycle arrest and improve its radiosensitivity by targeting cyclin D1/E1 [6]. Sequence analysis found that miR-16-5p is a potential target of CERS6-AS1, so this study speculated that CERS6-AS1 may target miR-16-5p to play a role in prostate cancer. Therefore, the purpose of this study is to analyze the expression of CERS6-AS1 and miR-16-5p in prostate cancer tissues and to explore the mechanism of CERS6-AS1 targeting miR-16-5p on the biological behavior of prostate cancer cells.

## 2. Materials and Methods

### 2.1. Materials

#### 2.1.1. Tissue Source

The prostate cancer tissues and adjacent tissues of patients with primary prostate cancer who underwent surgical resection in our hospital from January 2018 to October 2019 were collected. The average age was 62.0 ± 9.5 years. Inclusion criteria were as follows: primary prostate cancer diagnosed by histology; it was agreed to collect tumor tissues and paired adjacent tissues for research. Exclusion criteria were as follows: patients with other malignant tumors. This study was approved by the ethics committee of our hospital and conforms to the principles of the declaration of Helsinki. Written informed consent was obtained from each participant.

#### 2.1.2. Cells and Reagents

Human pancreatic cancer cell DU145 and human normal prostate epithelial cell RWPE-1 were purchased from the National Institutes of Health. Lipofectamine 2000 was purchased from Invitrogen company of the United States. PrimeScript™ reverse transcription reagent and SYBR Green Master Mix kit were purchased from Takara. CERS6-AS1's small interfering RNA (si-CERS6-AS1), small interfering RNA negative control (si-NC), miR-16-5p mimics, miRNA mimic negative control (MIR NC), miR-16-5p inhibitor (miR-16-5p inhibitor), and luciferase report intelligence were purchased from Sangong Bioengineering (Shanghai) Co., LTD. Cell counting Kit (CCK-8), Trizol reagent, goat anti-rabbit IgG secondary antibody, rabbit-derived HMGA2 polyclonal antibody, rabbit-derived glyceraldehyde phosphate dehydrogenase (GAPDH) polyclonal antibody were purchased from Proteintech; annexin V-FITC apoptosis detection kit was purchased from Beijing boasen company.

### 2.2. Method

#### 2.2.1. Cell Culture

DU145 cells and RWPE-1 cells were cultured in DMEM medium containing 10% fetal bovine serum and in 37°C incubator containing 5% CO_2_. When the cell density was 80%, the cells were digested with 0.25% trypsin and subcultured in the ratio of 1 : 3.

#### 2.2.2. RT qPCR Was Used to Detect the Expression of CERS6-AS1 and miR-16-5p in Prostate Cancer Tissues

Total RNA was extracted from prostate cancer tissues, adjacent tissues, DU145 cells, and RWPE-1 cells with Trizol reagent. The concentration and purity of total RNA were measured by UV spectrophotometer. When the ratio of A260/A280 was in the range of 1.8-2, the RNA was considered qualified. Take 1 *μ*g total RNA cDNA was synthesized by PrimeScript™ reverse transcription kit, and then, the cDNA was used as amplification template for RT qPCR by SYBR Green master mix. The relative expressions of CERS6-AS1 and miR-16-5p were calculated by 2^-*ΔΔ*CT^ method. miR-16-5p upstream primer 5′-TAGCAGCACGTAAATATTGGCG-3′, downstream primer 5′-TGCGTGTCGTGGAGTC-3′; U6 upstream primer 5′-CTCGCTTCGGCAGCACA-3′, downstream primer 5′-AACGCTT CACGAATTTGCGT-3′; CERS6-AS1 upstream primer 5′-GCAGCCCAGCAGAAGTAGGA-3′, downstream primer 5′-GAGCATAGGGAAGCAACTCTCAG-3′; GAPDH upstream primer 5′-CGAGCCACATCGCTCAGACA-3′, downstream primer 5′-GTGGTGAAGACGCCAGTGGA-3′.

#### 2.2.3. Cell Transfection and Grouping

A 24-well plate was taken, and 500 *μ*L medium containing 1 × 105 DU145 cells was added to each well, and transfection was carried out when the density was 40%. Use 50 *μ*L serum free medium diluted with 20 pmol RNA and recorded as solution A. Use 50 *μ*L serum free medium dilution 2 *μ*L liposome Lipofectamine 2000, recorded as liquid B. Gently mix liquid A and liquid B and let them stand for 5 min. Suck liquid B and add it to liquid A, flick it and mix it evenly, and place at room temperature for 15 min. During transfection, the 24-well plate medium was replaced with serum-free medium with 400 *μ*L per well. A/B complex was slowly added into the medium, shaken well, and incubated for 6 h. After serum-free medium was removed, the medium was changed to normal medium for further culture. Cells were collected and transfected for 48 h, RNA was extracted according to “1.2.2,” and the relative levels of CERS6-AS1 or miR-16-5P were detected by RT-PCR to detect the transfection effect. DU145 cells were divided into si-CERS6-AS1 group, si-NC group, miR-16-5P mimic group, miR-NC group, and si-CERS6-AS1+miR-16-5p inhibitor group according to different transfection vector or oligonucleotide experiments. Normal DU145 cells were recorded as the control group.

#### 2.2.4. The Proliferation of DU145 Cells Was Detected by CCK-8 Experiment

DU145 cells in each group were inoculated into 96-well plates at a density of 1 × 103 cells/well for 48 h after transfection, and 3 replicates were set. After cell adhesion, add 10 *μ*L CCK-8 solution to each well and continue to culture for 2 h. The absorbance (A) at 450 nm was measured by spectrophotometer. The experiment was repeated three times. Proliferation inhibition rate (%) = (control well A − experimental well A)/(control well A − blank well A) × 100%.

#### 2.2.5. Colony Formation Assay Was Used to Detect the Clonogenic Ability of DU145 Cells

DU145 cells in each group were inoculated into 6-well plates at a density of 1 × 103 cells per well after transfection of 48 h. The plates were slowly rotated to evenly disperse the cells, and the cells were placed in an incubator for incubation for 12-14 days, set in 3 repetitions. Change the medium every three days. When cell colonies were seen, the culture was terminated, and the colonies were fixed with methanol for 20 min and stained with 0.1% crystal violet for 20 min. The number of colonies with more than 50 cells was counted under an optical microscope. The experiment was repeated three times.

#### 2.2.6. Apoptosis of DU145 Cells Was Detected by Flow Cytometry

DU145 cells transfected for 48 h in each group were digested with 0.25% trypsin, and 1 × 105 cells were suspended in 500 *μ*L 1× binding buffer. Annexin V-FITC (5 *μ*L) and PI (5 *μ*L) were successively added to each group for fine staining. After 20 min of dark incubation, apoptosis rate of DU145 cells in each group was analyzed by flow cytometry.

#### 2.2.7. The Migration Ability of DU145 Cells Was Detected by Scratch Healing

DU145 cells, which had been transfected for 48 h, were inoculated with 6-well plates at a density of 1 × 106 cells/well by 0.25% trypsin digestion. When all cells are lined on the bottom of the plate, use 200 *μ*L pipette tip perpendicular to the whole plate to create cell scratches. The cell culture medium was aspirated, and the 6-well plate was rinsed with PBS three times, and then, the cell fragments were washed away. Serum-free medium was added, and the scratch width was measured at 0 h. The culture plate was put into the incubator for cultivation. After 24 hours of cultivation, it was taken out and photographed, and the width of scratch was measured for 24 hours. Scratch healing rate (%) = (0 h scratch width − 24 h scratch width)/0 h scratch width x 100%.

#### 2.2.8. The Expression of HMGA2 Protein in DU145 Cells Was Detected by Western Blot

RIPA buffer was lysed and transfected into DU145 cells in each group for 48 h. The cells were incubated on ice for 30 min and centrifuged at 12000 r/min at 4°C for 15 min to collect supernatant. Protein concentration was determined by BCA kit. 30 *μ*g cell protein was isolated by SDS-Page (100 V and 100 min), wetted (300 mA and 20 min) onto NC membrane, sealed with 5% skim milk at room temperature for 2 h, and then added with primary antibody of HMGA2 and GAPDH (diluted at 1 : 500 by volume ratio) for 12 h at 4°C and secondary antibody (diluted at 1 : 1000 by volume ratio) for 2 h at room temperature. The protein bands were colored with chemiluminescence kit. Image J software measured the gray values of HMGA2 and GAPDH strips, and the HMGA2 expression level was expressed by the ratio of HMGA2 and GAPDH strips.

#### 2.2.9. Double Luciferase Report Experiment

Wild-type (WT) CERS6-AS1 and HMGA2-3′-UTR fragments containing predicted miR-16-5P binding sites were synthesized and cloned into psiCHECK-2 reporter vector to construct wt-CERS6-AS1 and wt-HMGA2 luciferase reporter plasmids. Mutants (MUT) CERS6-AS1 and HMGA2-3′-UTR fragments were synthesized by point mutation kit and cloned into psiCHECK-2 to construct mut-CERS6-AS1 and mut-HMGA2 reporter plasmids, respectively. Logarithmic DU145 cells were inoculated with 6-well plates. When the cells grew to 50% and converged, Lipofectamine 2000 was used to cotransfect WT or MUT reporter plasmids with miR-16-5p mimics and miR-NC, respectively. After 48 h, the luciferase activity was determined by dual luciferase reporter gene assay system.

### 2.3. **S**tatistical Methods

SPSS 21.0 software was used for statistical analysis, and the data were expressed as mean ± standard deviation (x ± s). Independent sample *t*-test was used for the comparison between the two groups, and one-way ANOVA and *SNK-q* test were used for the comparison between the multiple groups. *P* < 0.05 was regarded as statistically significant.

## 3. Results

### 3.1. Expression of CERS6-AS1 and miR-16-5p in Prostate Cancer

RT-qPCR was used to detect the expressions of CERS6-AS1 and miR-16-5p. The results showed that the relative levels of CERS6-AS1 and miR-16-5p in prostate cancer tissues were significantly higher than those in adjacent tissues (*P* < 0.05). Compared with RWPE-1 cells, the relative level of CERS6-AS1 in DU145 cells increased significantly (*P* < 0.05), and the relative level of miR-16-5p decreased significantly (*P* < 0.05), see Figure 1.

### 3.2. Detection of CERS6-AS1 Expression after Silencing CERS6-AS1 Treatment

Compared with si-NC transfection, the relative levels of CERS6-AS1 in DU145 cells were significantly decreased after transfection of si-CERS6-AS1A, si-CERS6-AS1B, and si-CERS6-AS1C (*P* < 0.05), see Figure 2.

### 3.3. Effects of Silencing CERS6-AS1 on Proliferation, Apoptosis, and Migration of DU145

Compared with the control group and si-NC group, the relative level of CERS6-AS1, HMGA2 protein expression, colony formation number, and scratch healing rate of DU145 cells in si-CERS6-AS1 group decreased significantly (*P* < 0.05), while the relative level of miR-16-5p, proliferation inhibition rate, and apoptosis rate increased significantly (*P* < 0.05), see Figure 3 and Table 1.

### 3.4. Effects of Overexpression of miR-16-5p on Proliferation, Apoptosis, and Migration of DU145

Compared with the control group and miR-NC group, the relative level of miR-16-5p and proliferation inhibition rate and apoptosis rate of DU145 cells in miR-16-5p mic group were significantly increased (*P* < 0.05), and the expression of HMGA2 protein and colony formation number and scratch healing rate were significantly decreased (*P* < 0.05), see Figure 4 and Table 2.

### 3.5. Targeting Relationship between CERS6-AS1, miR-16-5p, and HMGA2

Starbase online prediction shows that there are complementary sequences between CERS6-AS1 and miR-16-5p, and targets online prediction shows that there are complementary sequences between miR-16-5p and HMGA2-3′-UTR, as shown in Figure 5. Compared with miR-NC and wt-CERS6-AS1 (or wt-HMGA2) cotransfection, the luciferase activity of DU145 cells cotransfected with miR-16-5p mimics and wt-CERS6-AS1 (or wt-HMGA2) decreased significantly. Compared with miR-NC and mut-CERS6-AS1 (or mut-HMGA2) cotransfection, there was no significant change in luciferase activity of DU145 cells after cotransfection of miR-16-5p mimics and mut-CERS6-AS1 (or mut-HMGA2), as shown in Table 3.

### 3.6. Inhibition of miR-16-5p Can Reverse the Effects of CERS6-AS1 on Proliferation, Apoptosis, and Migration of DU145 Cells

Compared with the control group, the relative level of miR-16-5p and proliferation inhibition rate and apoptosis rate of DU145 cells in si-CERS6-AS1 group were significantly increased (*P* < 0.05), and the expression of HMGA2 protein and colony formation number and scratch healing rate were significantly decreased (*P* < 0.05). Compared with si-CERS6-AS1 group, the relative level of miR-16-5p and proliferation inhibition rate and apoptosis rate of cells in the si-CERS6-AS1+miR-16-5p inhibitor group decreased significantly (*P* < 0.05), and the expression of HMGA2 protein and the number of colony formation and scratch healing rate increased significantly (*P* < 0.05), see Figure 6 and Table 4.

## 4. Discussion

lncRNA can affect the proliferation, apoptosis, metastasis, and invasion of prostate cancer cells, providing a potential target for inhibiting the occurrence and metastasis of prostate cancer [7]. This study analyzed the difference in CERS6-AS1 expression levels between prostate cancer, adjacent tissues, and normal prostate epithelial cells. The results showed that CERS6-AS1 was significantly upregulated in prostate cancer and prostate cell DU145. Relevant studies have shown that patients with pancreatic ductal carcinoma with high expression of CERS6-AS1 have a short overall survival time. Knockout of CERS6-AS1 can weaken the proliferation, migration, and invasion of pancreatic ductal carcinoma cells, induce apoptosis, and inhibit tumor growth in vivo [8]. The high expression of CERS6-AS1 in breast cancer can promote the proliferation of cancer cells and inhibit the apoptosis [9]. In this study, si-CERS6-AS1 was transfected for functional analysis. It was found that after silencing CERS6-AS1, the proliferation, clone formation, and migration of DU145 cells were inhibited, but the apoptosis rate increased, which was consistent with the anticancer effect of knockdown CERS6-AS1 reported by Yun et al. These findings suggest that CERS6-AS1 plays an oncogene role in prostate cancer, and silencing CERS6-AS1 may be a potential treatment strategy for prostate cancer.

Many studies have shown that lncRNA can eliminate the inhibitory effect of miRNA on its target genes by binding with miRNA, so as to play a regulatory role in the progression of prostate cancer. For example, lncRNA MEG3 can affect the proliferation, metastasis, and apoptosis rate of prostate cancer cells. This regulation depends on the regulation of miR-9-5p and its target gene QKI-5 [10]. lncRNA LOXL1-AS1 mediates the resistance of prostate cancer cells to adriamycin by upregulating EGFR expression by targeting miR-let-7a-5p [11]. Previous studies have shown that CERS6-AS1 can bind to miR-15a-5p and miR-125a-5p and function in pancreatic ductal carcinoma and breast cancer [9, 10]. miR-16-5p is a tumor suppressor. Studies have pointed out that upregulating the expression of miR-16-5p can inhibit the proliferation and metastasis of liver cancer cells [12]. miR-16-5p inhibits the survival of prostate cancer cells by targeting protein kinase 3 (AKT3), regulates cell cycle distribution, and induces apoptosis [13]. In addition, miR-16-5p also mediates the inhibitory effect of knockdown Linc0021 on the biological behavior of nonsmall cell lung cancer [14]. This study found that the expression of miR-16-5p was downregulated in prostate cancer tissues and DU145 cells and confirmed that miR-16-5p was negatively regulated by CERS6-AS1. The verification of the function of miR-16-5p showed that overexpression of miR-16-5p significantly inhibited the proliferation, clone formation, and migration of DU145 cells and promoted apoptosis, which was consistent with the anticancer effect of silencing CERS6-AS1.

Further exploration found that HMGA2 was a potential target of miR-16-5p. Studies have shown that HMGA2 expression is upregulated in prostate cancer, which is related to lymph node metastasis and Gleason grade. Downregulation of HMGA2 can inhibit proliferation, invasion, and migration and increase the rate of apoptosis [15, 16]. This study confirmed that miR-16-5p targeted negative regulation of HMGA2 expression, and silencing CERS6-AS1 significantly inhibited HMGA2 expression by upregulating miR-16-5p, suggesting that CERS6-AS1/miR-16-5p/HMGA2 axis may exist in prostate cancer. The response experiment showed that inhibiting the expression of miR-16-5p significantly reversed the effects of silencing CERS6-AS1 on the proliferation, apoptosis, migration, and HMGA2 expression of DU145 cells, which further indicated that the carcinogenic effect of CERS6-AS1 in prostate cancer was achieved at least in part by regulating the miR-16-5p/HMGA2 axis.

In conclusion, the expression of CERS6-AS1 is upregulated in prostate cancer, and silencing CERS6-AS1 can inhibit the proliferation and migration of DU145 cells and promote cell apoptosis. The mechanism is related to the upregulation of miR-16-5p/HMGA2 axis. These findings suggest that CERS6-AS1/miR-16-5p/HMGA2 axis may be a potential target for treatment of ovarian cancer before treatment.

## Figures and Tables

**Figure 1:** The expression level of CERS6-AS1 and miR-16-5p. (a). The expression level of CERS6-AS1 expression in prostate cancer. (b). The expression level of miR-16-5p. (c). The expression level of CERS6-AS1 expression in prostate cancer cells. (d). The expression level of miR-16-5p expression in prostate cancer cells.

**Figure 2:** The expression level of CERS6-AS1 in NC and si-CERS6-AS1 cells.

**Figure 3:** Effect of silencing CERS6-AS1 on DU145 apoptosis and HMGA2 protein expression.

**Figure 4:** Effect of overexpression of miR-16-5p on apoptosis and HMGA2 protein expression of DU145 cells.

**Figure 5:** Complementary sequences of CERS6-AS1 and miR-16-5p and miR-16-5p and HMGA2.

**Figure 6:** Inhibition of miR-16-5p can reverse the induction of apoptosis of DU145 by silencing CERS6-AS1 and the inhibition of HMGA2 protein.

**Table 1:** Effects of silencing CERS6-AS1 on proliferation, migration, and apoptosis of DU145 ($\bar{\text{x}}\pm \text{s}$, *n* = 9).

Group	CERS6-AS1	miR-16-5p	HMGA2	Inhibition rate (%)	Apoptosis rate (%)	Colony formation number	Scratch healing rate (%)
Control	1.00 ± 0.00	1.00 ± 0.00	0.73 ± 0.05	0.00 ± 0.00	6.86 ± 0.40	124.44 ± 3.50	68.85 ± 1.85
si-NC	0.99 ± 0.03	1.00 ± 0.04	0.74 ± 0.06	0.02 ± 0.02	6.93 ± 0.64	124.89 ± 5.28	68.95 ± 1.72
si-CERS6-AS1	0.24 ± 0.02^∗^^#^	4.13 ± 0.09^∗^^#^	0.27 ± 0.03^∗^^#^	56.77 ± 3.02^∗^^#^	22.73 ± 1.06^∗^^#^	67.00 ± 2.36^∗^^#^	36.46 ± 1.22^∗^^#^
*F*	3946.846	9089.907	278.100	3179.028	1261.434	654.922	1203.570
*P*	0.000	0.000	0.000	0.000	0.000	0.000	0.000

Note: Compared with control group, ^∗^*P* < 0.05; compared with si-NC group, ^#^*P* < 0.05.

**Table 2:** Effects of overexpression of miR-16-5p on proliferation, migration, and apoptosis of DU145 ($\bar{\text{x}}\pm \text{s}$, *n* = 9).

Group	miR-16-5p	HMGA2	Inhibition rate (%)	Apoptosis rate (%)	Colony formation number	Scratch healing rate (%)
Control	1.00 ± 0.00	0.75 ± 0.05	0.00 ± 0.00	7.10 ± 0.46	127.11 ± 4.51	68.21 ± 1.76
miR-NC	1.01 ± 0.02	0.75 ± 0.06	0.01 ± 0.02	6.93 ± 0.47	127.33 ± 3.65	66.82 ± 2.26
miR-16-5p mimic	5.43 ± 0.12^∗^^#^	0.14 ± 0.01^∗^^#^	65.88 ± 2.73^∗^^#^	26.08 ± 0.84^∗^^#^	52.33 ± 1.49^∗^^#^	27.40 ± 1.11^∗^^#^
*F*	11907.182	540.145	5240.047	2874.495	1406.721	1536.028
*P*	0.000	0.000	0.000	0.000	0.000	0.000

Note: Compared with control group, ^∗^*P* < 0.05; compared with miR-NC group, ^#^*P* < 0.05.

**Table 3:** Double luciferase report experiment ($\bar{\text{x}}\pm \text{s}$, *n* = 9).

Group	wt-CERS6-AS1	mut-CERS6-AS1	wt-HMGA2	mut-HMGA2
miR-NC	1.00 ± 0.08	1.01 ± 0.06	1.01 ± 0.09	1.04 ± 0.09
miR-16-5p	0.25 ± 0.02^∗^	1.04 ± 0.08	0.33 ± 0.02^∗^	0.99 ± 0.07
*t*	27.285	0.900	22.127	1.316
*P*	0.000	0.381	0.000	0.207

Note: Compared with miR-NC group, ^∗^*P* < 0.05.

**Table 4:** Inhibition of miR-16-5p can reverse the effect of silencing CERS6-AS1 on proliferation, migration, and apoptosis of DU145 ($\bar{\text{x}}\pm \text{s}$, *n* = 9).

Group	miR-16-5p	HMGA2	Inhibition rate (%)	Apoptosis rate (%)	Colony formation number	Scratch healing rate (%)
Control	1.00 ± 0.00	0.74 ± 0.06	0.00 ± 0.00	6.88 ± 0.60	124.89 ± 5.82	69.04 ± 2.59
si-CERS6-AS1	4.14 ± 0.13^∗^	0.27 ± 0.03^∗^	56.81 ± 3.55^∗^	22.71 ± 0.93^∗^	66.00 ± 2.75^∗^	36.70 ± 0.84^∗^
si-CERS6-AS1+miR-16-5p inhibitor	1.58 ± 0.09^#^	0.61 ± 0.04^#^	15.30 ± 0.93^#^	11.33 ± 0.53^#^	109.22 ± 4.08^#^	59.97 ± 2.06^#^
*F*	3014.928	260.705	1732.365	1195.066	432.445	644.519
*P*	0.000	0.000	0.000	0.000	0.000	0.000

Note: Compared with control group, ^∗^*P* < 0.05; compared with si-CERS6-AS1 group, ^#^*P* < 0.05.

## Data Availability

The data used to support this study are available from the corresponding author upon request.
